The article "Construction of Network Ideological and Political Management Platform in Institution of Higher Learning Based on Information Technology under the New Media Environment" was retracted in 2023. Reasons: unreliable results or conclusions; lack of ethics approval or compliance; concerns about the data; concerns about the results or conclusions.

# Construction of Network Ideological and Political Management Platform in Institution of Higher Learning Based on Information Technology under the New Media Environment

**DOI:** 10.1155/2022/3794354

**Published:** 2022-08-31

**Authors:** Xingchen Li

**Affiliations:** Civil Aviation Flight University of China, Flight Technology College, Guanghan, Sichuan 618300, China

## Abstract

The resources used by network ideological and political educators to achieve their goals make up the entire collection of materials and components that make up network ideological. Some academic institutions, such as Nanjing University of Aeronautics and Astronautics, rely on new media to develop novel ideological techniques, such as “Xuchuan's political work practices,” which have had a significant impact on young college students. WeChat, Weibo, and Twitter are just a few of the new media platforms that have emerged as a result of China's ongoing process of digitalization. The development of new media information technology has subtly altered how political and ideological management is conducted in academic institutions. This study of the network ideological in higher education institutions is based on information technology and the new media environment. The study reveals that the highest rate of knowing very well is 14.36%, and the highest rate of knowing well is 25.65%, according to the trend of understanding new media information technology. Only 3.35% said they were unsure. According to the experiment, there is a rising trend in understanding and understanding unity as the number of samples increases. In this instance, it makes sense to use new media to advance the ideological goals of a higher education institution. The network ideological and political management platform of the institution of higher learning uses information technology to support online discussion and analysis, which is crucial for fostering students' ethical values and a healthy way of thinking.

## 1. Introduction

The primary channel and setting for college students to engage in Marxist theory education and network ideology in institutions of higher learning is the main classroom that serves as a resource for helping students develop the right worldview, outlook on life, and values. Ideology is a systematic project that runs throughout a person's entire developmental process, beginning with morality and society in primary school, ideology and morality in junior high school, ideology and politics in senior high school, and fundamentals of Marxism in the final university. Its goal is to improve people's capacity for understanding and affecting change in the world [1]. Online ideological resources are the sum of various materials and elements developed and utilised by ideological and political educators to achieve the purpose of online ideological. Some institutions of higher learning, such as Nanjing University of Aeronautics and Astronautics, rely on new media to innovate new methods of ideological such as “Xuchuan's ideological and political work method.” It has generated strong repercussions among young college students [2]. In terms of educational effect, with the popularization of the network and the construction of campus network, college students have more different views to contact and understand through the network, and their thoughts and behaviors are increasingly developing in the direction of personalization. In this case, it is difficult for them to passively accept various concepts instilled by teachers as before, and the dominant position of teachers is affected, which also weakens the effect of network ideological. With the continuous improvement of China's opening to the outside world and the openness of the Internet, various nonsocialist thoughts and the concepts of different countries and nations in our exchanges with different countries continue to impact the content of our traditional online ideological. The dominant position of socialist core values and other mainstream values is affected, resulting in the phenomenon of “worshiping foreign countries and fawning on foreign countries” of college students from time to time [3, 4].

The public, especially college students, now primarily obtains information through new media, which is rapidly evolving and developing and producing an endless variety of new media forms. The new media era is embracing people and society with this new mindset, and ideological and political educators in institutions of higher education on the cutting edge of online ideological education are destined to face the wave, catch up with it, and surpass it on the way. The environment and circumstances of network ideological have changed under the new information technology situation. The network ideological in institutions of higher education must also adapt to the times, take advantage of the global opportunity presented by the rapid development of information technology, and continually look for new models, new approaches, and new techniques for network ideological and political courses in institutions of higher education [5, 6]. The development of Chinese education is also heavily influenced by network ideological and political teaching, which has profound implications and outlooks on the world. Higher education institutions must actively use network new media technology to properly guide students if they want to better penetrate the network ideological. In today's higher education institutions, the method of information transmission also takes the form of a hierarchical scattering. The school's administrative centre is one component of a complex system, and each college consists of a number of subsystems. In addition, because of the diversity and speed with which new media technologies disseminate information, it is simple for tight controls on new media to become loosened. As a result, a lot of unfavorable information demoralises college students and harms the advancement of their education.

The application scope of network new media in network ideological has been significantly expanded, which also benefits from the unique advantages of network new media itself. For example, online new media can strengthen the attraction of ideological to college students; the application of network new media can standardize students' words and deeds and improve students' quality; with the help of network new media, we can create a perfect network ideological and political management platform in institution of higher learning [7]. The construction of network ideological and political management platform in institution of higher learning provides more ways and methods for network new media information transmission. The play of the efficiency of the network platform itself can bring more help and support to the information transmission of new media information technology. It speeds up the construction and expansion of the carrier of network ideological on the network ideological and political management platform of institution of higher learning, keeps the network ideological from being affected by the new situation and steadily advance, advocates the educational concept to conform to the development of the times and keep pace with the times, and improves the application ability and media literacy of educational subjects and objects to new media [8]. In addition, based on information technology, on the network ideological and political management platform of institution of higher learning, we can quickly understand social hot issues and carry out online discussion and analysis according to these contents, which plays an important role in the formation of students' good values and the cultivation of correct thinking system [9].

The innovations in this study are as follows:

1. This study builds the network's ideological and political management platform's system structure diagram. An information platform is built with information and network technology that is tightly integrated with other systems of the campus network and connected to the Internet and can carry out the functions of interactive teaching between teacher and student, publicity, consultation, and communication, monitoring, and effective management of the online ideologies of college students.
2. This study analyzes the organizational teaching using new media informatization and constructs a simplified data flow diagram of student users in this study. In the process of database design, the document describing various basic elements stores the description of the database and its table structure. Its function is to give specific meaning to each component in the data flow diagram and provide an accurate and unambiguous description and description for the system elements.

## 2. Related Work

The research on the informatization of network ideological in institution of higher learning has become a new problem before us. We need to deeply study the current environment of network ideological with a scientific attitude and analyze the characteristics of information society and what impact this information society has on network ideological in institution of higher learning and how to use scientific theories and educational concepts to promote the smooth development of informatization of ideological will become new issues to be solved.

### 2.1. Research on Network Ideological in Institution of Higher Learning

Lili et al. think that although the school is actively building a digital campus and has certain informatization conditions, so far there is no complete network ideological information system, and even in the process of applying informatization, the above problems exist to varying degrees, and the overall application level of network ideological informatization is low [10]. Cao analyzes the present situation, predicament, and future of network ideological in institution of higher learning from the perspective of globalization and thinks that the five major dilemmas of network ideological in institution of higher learning are low completion rate, high requirements for teachers, high requirements for technical support, unsatisfactory acceptance effect, and difficulties in evaluation and testing [11]. Heng-Zhao et al. believe that the massive open online course curriculum is generated through the communication, discussion, and sharing of participants, and it integrates social networks, experts in a certain field, and resources available online through various forms of social media. Thus, in the early foreign literature of massive open online course, the characteristics of “online learning” and “student gathering” in massive open online course were mainly emphasized [12]. Hua et al. proposed that teachers should set up a teaching mode of teacher-student interaction in the online ideological and political classroom and encourage students to freely discuss social and political events, which can deepen students' knowledge consolidation and improve students' attention to social and political events [13]. Chen et al. show that the network ideological in institution of higher learning is mainly aimed at college students, and counselors should rely on the new media network platform to pay attention to college students' state of mind at any time, so as to guide and supervise students' thoughts [14]. Huang et al. show that the educational content is divorced from reality and influenced by the convenient conditions of informatization. Many college teachers may ignore the interests of the educated themselves and other situations in the process of ideological on the Internet, resulting in superficial “innovation” in educational content that is divorced from reality [15]. Chen et al. showed that college teachers should cultivate students' ability to analyze political events through students' talk about events, guide students to correctly understand the essence of events, and establish correct outlook on life and values for college students [16]. Zhu et al., on the basis of analyzing the reasons, advantages, and disadvantages of the rise of massive open online course, discussed that massive open online course has a positive effect on the popularization and internationalization of higher education and the reform of teaching methods. From the perspective of platform construction in massive open online course, it is concluded that the diversified platform development in massive open online course can support the reform of blended teaching in schools [17]. Rong proposed that institution of higher learning should implement the teaching mode of “two micro-one-end” in online ideological and political courses, which was conducive to the establishment of a harmonious teacher-student relationship [18]. Li et al. proposed that the digital campus construction plan has a special financial budget, so the construction of the information platform for ideological can rely on the hardware equipment formed by the digital campus construction. It is only necessary to ensure that the software construction can be organically integrated with the digital campus, so it has strong economic feasibility [19].

### 2.2. Research Methods Proposed in This Study

A more recent form of media development is new media. It first appears on the foundation of the increasingly sophisticated information technology, such as the microcomputer, network, and intelligent terminal, and has developed into a significant means of communication and information dissemination. Higher education institutions play a significant role in developing Chinese socialist builders and successors. They incorporate social information resources into information technology, actively develop and fully utilise modern information technology, apply modern information technology guidance to all areas and processes of contemporary education and teaching, fully utilise information technology from wholesome and scientific information on the network, educate college students, and enhance their overall quality. Ideological and political workers can receive information immediately, thanks to the ideological and political management platform's timeliness. The new media network platform's information content is comprehensive, covers a wide range of topics, has no national borders, and can swiftly spread and share information from all over the world. This information can broaden college students' perspectives and create a collision of cultural ideas and values, as well as increase productivity.

With its timeliness, interactivity, openness, and other characteristics, information technology [20, 21] provides a new platform for network ideological, which makes network ideological more vibrant and dynamic. This means of informatization synchronized with the times has a profound and long-term impact on the ideological and political work on the Internet. The space of ideological on the Internet has been expanded under the characteristics of openness and interactivity of informatization. Compared with the complex society, the university campus is a relatively closed pure land isolated from the world. The influence of the informatization of network ideological has created very favorable conditions in the acquisition channels and methods of network ideological information and has been improved and expanded.

## 3. Research Method

### 3.1. Construction of Network Ideological Information Platform of New Media

Because network ideological activities are unique, building a platform for network ideological informatization among college students—a crucial step in the informatization of education—involves more than just solving technical issues. It also involves addressing how “people” will use the technology. This study analyzes the needs of the system, focusing on the work of relevant personnel, the functional requirements, composition, and nonfunctional requirements of the current network ideological information platform in institutions of higher learning, according to the possible development direction in the future, and combined with the actual situation of the network ideological in Shandong Vocational College of Tourism. However, the new media platform has the characteristics of virtuality, and there are also some shortcomings in the construction of Chinese laws and regulations in this area. New media is an important medium for students to obtain information and disseminate information. This causes numerous issues with the management of the network platform and the release of information. On the network, there is a lot of offensive information and misinformation. However, because they lack social experience and mental maturity, college students are more susceptible to being influenced by false information. An information platform is built with information and network technology that is tightly integrated with other systems of the campus network and connected to the Internet and can carry out the functions of interactive teaching between teacher and student, publicity, consultation, and communication, monitoring, and effective management of the online ideologies of college students. The network ideological and political management platform system's functional structure is depicted in Figure 1 due to the network ideological's universality, diversity of ways and methods, and complexity of the education process, as well as the relevant personnel's work within the system and the system's overall functional requirements.

The information platform system of ideological is divided into the following four subsystems:

#### 3.1.1. Network-Based Subsystem of Political and Ideological Instruction

By building a network course teaching system, we can implement network instruction. The subsystem is divided into teacher work modules and student learning modules based on the various activities that teachers and students engage in.

#### 3.1.2. Network Propaganda Subsystem for Ideology and Politics

On the Internet, ideological and political propaganda should adhere to a set of principles and guiding ideologies, namely, accurate reporting of true information, advice for uncertain information, and ardent promotion of accurate information.

#### 3.1.3. Network Consultation and Communication Subsystem for Ideologies and Politics

College students can consult with full-time ideological and political teachers or other experts and teachers anonymously on the platform for many secret topics that college students do not want to discuss out loud, such as emotional distress, interpersonal barriers, sex education, and schizophrenia.

#### 3.1.4. Network Ideological and Political Monitoring Subsystem

While propagating positive information, we should also try our best to block the negative information's influence on students through various measures and try our best to prevent students from directly contacting bad moral education information, such as monitoring the content of network information, making relevant statistics by administrators, timely feeding back information to relevant departments, and establishing early warning mechanism [22].

Schools should assist college students to use new media reasonably, guide them to absorb healthy information, and eliminate the negative effects of bad information on college students' behaviors and thoughts in time. It can also better show the unique advantages of new media, enable students to grasp the social development trends more comprehensively and accurately, standardize students' behaviors, and strengthen students' quality construction. The students' answers to the exercises are independent, so the conditions of the answer results of the students' Tao exercises are distributed as follows:

(1) $$\begin{array}{c} L\left(A_{i}|C_{i}\right)=\prod_{j=1}^{m}P\left(1-P_{ij}\right). \end{array}$$

For *I* students, the answer results are distributed as follows:

(2) $$\begin{array}{c} L\left(A|C\right)=\prod_{i=1}^{I}L\left(A_{i}-C_{i}\right). \end{array}$$

Next, in order to solve the parameters *t*_*j*_ and *l*_*j*_, we first get the edge distribution of the answer result as follows:

(3) $$\begin{array}{c} L\left(A\right)=\prod_{i=1}^{I}L\left(A_{i}\right)=P\left(A_{i}|C_{l}\right). \end{array}$$

In order to get the maximum likelihood estimation better, we take logarithms on both sides of the above formula:

(4) $$\begin{array}{c} \ln\;L\left(A\right)=L\left(A_{i}\right)=\sum_{i=1}^{l}. \end{array}$$

Then, the derivation of parameters *t*_*j*_ and *l*_*j*_ is obtained as follows:

(5) $$\begin{array}{c} \frac{\partial \;\ln L}{\partial t_{j}}=0\left(1\leq j\right),\\ \frac{\partial \;\ln L}{\partial l_{j}}=0\left(1\leq j\right). \end{array}$$

This is also a nonlinear equation system with unknown numbers. To solve the equations, we can use Newton–Raphson iteration method to get the numerical approximate solution.

Teachers, students, educational administration, and other relevant departments can all benefit from two-way interactive communication modes enabled by information technology, which can help with communication timeliness and frequency, education guidance, and the replacement of the previous teacher-led “force-feeding” education mode. Personalized guidance is provided to each student in collaboration with the teacher, guiding them to choose their own courses and topics in accordance with their personalities and goals, and fostering their overall well-being [23].

### 3.2. Effective Strategies for Promoting the Network Ideological in Institution of Higher Learning

#### 3.2.1. Change Teachers' Understanding of New Network Media

In college ideological, the application of new online media has become the mainstream trend. In order to comply with the development trend, teachers should change their understanding of new online media, fully understand and master online thinking and language, promote the team building of student cadres, build a platform for ideological of new online media, and use information technology to organize teaching. New media is closely related to the development of the times. Nowadays, in ideological in many institutions of higher learning, due to the limitation of teachers' thoughts and ages, they cannot correctly understand new media and learn new things on their own initiative, and some teachers even have resistance, which is not conducive to the application of new media technology in network ideological. After the emergence of information technology under the background of new media, its learning style has been changed, teachers' educational resources are more abundant, and interactive learning can be realized [24, 25]. Classroom is the main position of traditional education in institution of higher learning, and teachers need to face students with different learning foundations. In terms of curriculum arrangement and content explanation, the overall level of students in the class will be taken as a reference, which makes it difficult for students with unsatisfactory acceptance ability to adapt to classroom teaching progress, and knowledge points are omitted.

The rise of new media, which has many advantages, has also brought new thorny problems to the network ideological in institution of higher learning, including fierce competition in the higher education market and severe employment situation of teachers, and put forward new requirements for the network ideological. These problems cannot be effectively solved by traditional methods alone, which requires the government, schools, and ideological and political educators to make correct judgments and choices in theory and practice according to the characteristics of ideological advancing with the times. With the rapid development of information technology and the rapid popularization of new media, teachers think that college students' dependence on new media is no longer a simple spiritual dependence. They use information technology to hand in homework, check information on the Internet, and check calendars, maps, and other practical needs through mobile phones. More accurately, they should regard the Internet as a tool for learning and living. In order to change the present situation and show the application advantages of new media ideological, institutions of higher learning need to correctly understand the new network media in the process of education and teaching and encourage teachers to take the initiative to learn and apply information technology. In-depth research on the new features, new ways, new carriers, and new methods of network ideological in institution of higher learning in the new media era of teachers can make network ideological more in line with the development and laws of the times and better meet the vitality and requirements of the times.

#### 3.2.2. Make Full Use of New Media Informatization to Organize Teaching

In order to keep up with the pulse of the times and actively use cutting-edge educational technology for development, online ideological should actively try the construction method of online open courses, revitalize the existing online ideological and political teaching resources, and form a “problem-based” teaching logic based on the teaching principle of “students first, learning first” in terms of teaching organization, so as to promote the mutual promotion between teachers' teaching and students' learning, “In class” and “out of class” are interconnected, and “online” and “offline” are interconnected, which turns the knowledge system of traditional textbooks to the problem logic and cognitive logic of teaching. The innovation of network ideological methods also requires the continuous accumulation of information. Informatization is a way, procedure, and practice for people to understand and transform the world. The method is essentially an operable rule created by individuals based on their understanding of the real world in action, a way of thinking for particular practical applications, and a unique informational sequence. The description of the database and its table structure is stored in the document describing various basic elements as part of the database design process. Its purpose is to provide an accurate and unambiguous description of the system elements as well as specific meaning for each element in the data flow diagram. As seen in Figure 2, the following is an illustration of a student user's condensed data flow diagram and related data dictionary entries.

Faced with the emergence of information technology, our previous network ideological methods are facing a great test, which requires us to flexibly use the network ideological methods and be a conscientious person. At the same time, we should also aim at educators and ask them to find ways to improve themselves and their work, so that we can adjust and improve our work in time and enhance the effectiveness of our work. Let us assume that the probability that students are correct in exercises is as follows:

(6) $$\begin{array}{c} P_{ij}=a_{j}+\frac{1-a}{1+e^{-1.7\beta }}, \end{array}$$

*P*_*ij*_ indicates the correct probability of students in exercises. The larger the value, the higher the correct probability. *a*_*j*_ indicates the probability that the exercises are guessed correctly without any knowledge, and *β* indicates the discrimination degree of exercises *j*. The greater the discrimination degree, the better the students' true level can be distinguished. *a* indicates that the value is generally 0.25 in objective questions and 0 in subjective questions.

This representation is more convenient for the following calculation. The new probability formula is as follows:

(7) $$\begin{array}{c} P_{ij}^{Aij}=\left(1-P_{ij}\right). \end{array}$$

Assuming there are *J* exercises, the maximum likelihood function is constructed as follows:

(8) $$\begin{array}{c} L\left(\beta_{j},y_{j},D\right)={\left(1-P_{ij}\right)}^{1-Aij}. \end{array}$$

For the convenience of derivation, the corresponding log-likelihood function is generally considered:

(9) $$\begin{array}{c} \ln\;L=A_{ij}\ln\;P_{ij}+\left(1-A_{ij}\right). \end{array}$$

Then, the derivative of the processed maximum likelihood function about unknown parameters is derived, and the derivative is equal to 0:

(10) $$\begin{array}{c} \frac{\partial \;\ln L}{\partial \beta_{j}}=0\left(1\leq j\right),\\ \frac{\partial \;\ln L}{\partial y_{j}}=0\left(1\leq j\right). \end{array}$$

This is a nonlinear equation system with unknown numbers. By solving the equations, we can get the desired result.

The key component to guaranteeing the network ideology goal's impact is also its means. Effective ideology should satisfy the basic information needs of the populace, removing any doubts they may have about the ideology and providing them with certainty through the dissemination of diverse and scientific information.

Using new media information technology, through the network ideological and political management platform, video, audio, pictures, slides, and other forms will vividly present boring ideological and political content to students, so that students can deeply understand the connotation of ideological and guide them to establish correct ideological consciousness and political beliefs. The discourse platform theory of ideological in institution of higher learning is a comprehensive concept formed by combining theoretical knowledge of many disciplines, and the concept and characteristics of new media context are the important background and basis for defining it. Under the platform of network ideological and political management, students are guided to sublimate to the level of firm ideals, beliefs, and world outlook, and the ability to analyze and solve ideological and theoretical problems is coordinated with practical problems, so as to improve their cognitive ability and practical ability of scientific theory. In a word, the application of network ideological and political management platform under information technology in ideological and political work in institution of higher learning is the embodiment of student-oriented teaching concept, which is conducive to giving full play to the dominant position of college students in ideological, promoting the continuous improvement of students' innovative ability and practical ability, building a harmonious ideological and political work environment for college students, and having positive significance for the follow-up network ideological and political work development and reform and innovation.

## 4. Simulation Experiment and Analysis

The emergence of new media information technology allows teachers and students to communicate equally, but because of the screen, educators cannot observe students' expressions, actions, and activity status, which hinders the targeted development of online ideological.

As shown in Figure 3, 45.85% of the students think it is “good,” 17.14% of the students think it is “average,” and more than half of the students think that teachers' awareness of using new media should be strengthened. The arrival of the new media era has brought higher requirements to the teaching ability of educators, urging educators to keep learning and keep up with the development trend of education.

With the continuous development of information technology, QQ, Weibo, and social networking sites are also new media forms that students pay close attention to and use. With the development of smartphones, PC clients and mobile clients are interconnected, and mobile phones and the Internet are integrated in an all-round, timely, and convenient manner. In the investigation of the main uses of new media information technology, the distribution of the main uses of new media was investigated. Experiments were carried out in the categories of instant messaging, network public opinion, and entertainment. The experimental results are shown in Figure 4.

As shown in Figure 4, instant messaging takes the lead with a maximum of 93.15%, indicating that the new media provides a more convenient communication platform for college students, and students have a higher yearning for a broad field of communication. Institution of higher learning should make rational use of this to guide the formation of a communication circle that is more conducive to students' growth. The functions of entertainment and online public opinion can fully mobilize students' interest in learning, but it is also necessary to prevent the negative impact of excessive entertainment on students.

The living conditions in schools are limited, the frequency of TV and radio is not high, and the network can completely replace it; in addition to class, most students will choose to use mobile phones or computers to finish reading paper media. However, due to the influence of new media information technology, college students are prone to inertia thinking and dependent thinking. Although the network is full of information, it is also full of good and evil people, which has shaken the minds of college students. This requires our network ideological and political educators in institution of higher learning not to ignore the positive role of traditional media such as newspapers and magazines. The experiment was conducted in the form of TV, mobile phone, and Internet media, and the distribution of media usage is shown in Figure 5.

As shown in Figure 5, among the three media, the Internet accounts for the highest proportion, with an average of 45.13%, followed by mobile phones, with an average of 35.65%. At the bottom of the list is television, accounting for only 9.72% on average. This wide gap shows that in the life of college students, the use of new media information technology with mobile phones and the Internet as the main body has been very common in life. In the system, while realizing data sharing, the table is simplified to the greatest extent, the pertinence of the table is enhanced, data redundancy is reduced, and the running load of the database server is reduced to a certain extent. The system has established four data tables, which respectively record the data required in each module, including user information, basic student information, and teaching course information, as listed in Tables 1–3.

With the deepening of college students' informatization education, new media informatization technology has been widely used and gradually understood by college students. According to the investigation of the understanding of new media informatization technology, we get very familiar with, understand, and do not understand the three options for experimental analysis. The experimental results are shown in Figure 6.

As shown in Figure 6, according to the trend of understanding of new media information technology, the highest level of understanding can reach 14.36%, and the highest level of understanding can reach 25.65%; only 3.35% chose not to know. It can be found from Figure 6 that with the increase of the number of samples, there is an upward trend in understanding and understanding unity, which shows that college students now have the basic quality of using new media. In this case, it is a reasonable time to use new media to promote college online ideological.

New media information technology provides path reference for improving the effectiveness of college network ideological. This experiment divides the categories into less than 1 hour, 1−2 hours, and 2−5 hours to carry out the experiment. On this basis, this study puts forward the path of the application of new media information technology in college ideological and provides method support and reference for improving the effectiveness of college network ideological. The experimental analysis is carried out on “the change in the duration of using new media information technology every day.” The experimental results are shown in Figure 7.

As shown in Figure 7, students use new media information technology for a long time every day, and the average number of students who use 1–2 hours every day accounts for 5.58%; the average number of students who use 2–5 hours a day is 23.06%; the average number of students who use more than 5 hours a day is 25.91%.

## 5. Conclusions

The network ideological itself is a complex systematic project, and the individualized characteristics of the ideological also determine that the core of the information platform lies in people's use of information technology. Therefore, many problems often occur during the construction of the information platform, which cannot be accomplished overnight. Other unrealized parts of the system and other details need to be further enriched and improved in the future implementation process. In this study, based on the information technology in the new media environment, the network ideological in institution of higher learning has been studied. The research shows that according to the trend of understanding the new media information technology, the highest rate of knowing very well is 14.36%, and the highest rate of knowing well is 25.65%. Only 3.35% chose not to know. From the experiment, it can be found that with the increase of the number of samples, there is an upward trend of understanding and understanding unity. In this case, it is a reasonable opportunity to use new media to promote ideological in institution of higher learning. On the basis of summarizing the theoretical experience of predecessors, this study expounds on the theory of network ideological in institution of higher learning. Information technology has a profound influence on college students' ideology, value orientation, and life attitude. In view of the information age, this study makes a profound analysis of the problems of network ideological in institution of higher learning. Finally, from the informatization construction of educational subject and educational object, the network ideological and political management platform of institution of higher learning is constructed, and the informatization supervision of institution of higher learning is strengthened. As one of the important technologies for exporting Chinese culture and soft power, information technology should go further and further to expand its influence after its continuous development.

## Figures and Tables

**Figure 1:** System structure diagram of network ideological and political management platform.

**Figure 2:** Simplified data flow diagram of student users.

**Figure 3:** Survey of teachers' awareness of using new media.

**Figure 4:** Changes in the distribution of main uses of new media.

**Figure 5:** Distribution of media usage.

**Figure 6:** Trend of new media understanding.

**Figure 7:** Changes of students' time using new media.

**Table 1:** User information table.

Field	Description	Length	Type	Principal linkage
Id	User name	7	Int	Yes
Psd	Password	31	Char	
Name	Full name	14	Char	

**Table 2:** Basic information of students.

Field	Description	Length	Type	Principal linkage
Id	Student number	7	Int	Yes
Name	Full name	14	Char	
Age	Age	5	Int	
Depart	Faculty	21	Char	

**Table 3:** Teaching course information.

Field	Description	Length	Type	Principal linkage
PPTID	Courseware number	7	Int	Yes
Uid	User ID	7	Int	
Pptnum	Number of courseware	5	Int	
Pptpswd	Courseware password	11	Vachar	

## Data Availability

The data used to support the findings of this study are available from the author upon request.
